# Ten Hotspot MicroRNAs and Their Potential Targets of Chondrocytes Were Revealed in Osteoarthritis Based on Bibliometric Analysis

This article has been retracted.

**DOI:** 10.1155/2022/8229148

**Published:** 2022-04-09

**Authors:** Wei-Shang Hu, Qi Zhang, Si-Hui Li, Shuang-Chun Ai, Qiao-Feng Wu

**Affiliations:** ^1^Acupuncture and Moxibustion College, Chengdu University of Traditional Chinese Medicine, Chengdu, Sichuan, China; ^2^Chongqing Traditional Chinese Medicine Hospital, Chongqing, China; ^3^Mianyang Hospital of Traditional Chinese Medicine, Mianyang, Sichuan, China; ^4^Institute of Acupuncture and Homeostasis Regulation, Chengdu University of Traditional Chinese Medicine, Chengdu, Sichuan, China; ^5^Acupuncture & Chronobiology Key Laboratory of Sichuan Province, Chengdu, Sichuan, China

## Abstract

**Background:**

Osteoarthritis (OA) is one of the most common joint disorders and debilitating diseases. Current evidence suggests that microRNAs (miRNAs) play a critical role in the pathogenesis of OA and have great potential as new biomarkers and therapeutic targets. We aimed to analyze the trends and research status on miRNAs in OA and further demonstrate the hotspot miRNAs in OA via CiteSpace and VOSviewer.

**Methods:**

Publications regarding miRNAs and OA were extracted from the Web of Science (WOS) database on October 30, 2021. We assessed the number of publications, institutions, countries, authors, journals, cited references, and keywords with the help of the software tools CiteSpace and VOSviewer.

**Results:**

A total of 1109 articles were included. Research related to miRNAs and OA began to appear in 2008, and the overall trend is increasing. Chinese institutions have a leading advantage in the number of publications but lack high-quality and high-cited research and are laggard in co-cited literature. Ten miRNAs including miR-140, miR-146, miR-34, miR-181, miR-27, miR-9, miR-29, miR-21, miR-26, and miR-155 and chondrocytes were revealed as the most obvious miRNAs and a potential target for OA based on bibliometric analysis. More focus will be placed on a comprehensive study on chondrocytes regulated by miRNAs, which may accelerate possible diagnostic biomarkers and diagnostic biomarkers of OA in the future.

## 1. Introduction

Osteoarthritis (OA) is the most common joint disease, affecting an estimated more than 300 million people worldwide, and the increase of the age-standardized prevalence and annual incidence rate was 9.3% and 8.2%, respectively, from 1990 to 2017 [1–4]. With the increase of population aging and obesity, as well as the change of lifestyle, the prevalence of OA has also increased, and it has gradually become a joint disease that has the greatest impact on the quality of life of middle-aged and elderly people [3, 5]. The etiology of OA remains enigmatic, which may involve genetic susceptibility, metabolism, trauma, inflammation, biomechanics, aging, epigenetics, and other factors [2, 6]. Researchers have attempted to intervene in the out-of-control molecular pathways of OA in recent years, including bisphosphonates, catabolic enzymes targeting articular cartilage degradation, inducible nitric oxide synthase (iNOS), and NF-*κ*B inhibitors, but the experimental and clinical effects are not ideal [7, 8]. The main clinical treatments for OA are still limited to physiotherapy, NSAIDs, and eventual arthroplasty [9].

MicroRNA (miRNA) is a type of endogenous noncoding small RNA [10]. It affects the regulation of gene expression by degrading or inhibiting target gene mRNA translation to control target gene expression [11]. Current studies have established the role of miRNAs in regulating gene expression in articular chondrocytes and their significance to the pathogenesis of OA [12, 13]. Methods for maintaining or suppressing the expression of critical miRNAs involved in the pathogenesis of OA have the potential to find new diagnostic and therapeutic targets [12]; Zhang et al. [14]. However, there are more than 100 miRNAs found differentially expressed in OA cartilage [15]; Nugent [16]. Therefore, investigating the current research status, hotspots, and frontiers of miRNAs in OA is meaningful and necessary.

This study focused on the network of authors, countries, and institutions, as well as the analysis of co-cited references, co-occurring keywords, cluster analysis, and keyword burst, to explore the global trends and hotspots of the past research on miRNAs in OA. And further this study excavates the hotspot miRNAs, related mechanisms, and targets to provide a reference for follow-up research.

## 2. Methods

### 2.1. Search Strategy

Data were collected from the Science Citation Index Expanded (SCI-E) of the Web of Science Core Collection (WoSCC), including Science Citation Index Expanded (SCI-EXPANDED), Conference Proceedings Citation Index-Science (CPCI-S), Current Chemical Reactions (CCR-EXPANDED), and Index Chemicus (IC). The data retrieval strategy included the topic “microRNAs or miRNAs or microRNA or miRNA” and the topic “osteoarthritis”. Publication type and language had no restriction. The search year is limited to 1900 to 31 October 2021. WoS export information function is used to download the information including the author, affiliation, title, abstract, keywords, journal, publication year, WoS category, and citation of each publication.

### 2.2. Visualization Analysis Based on CiteSpace and VOSviewer

CiteSpace 5.8.R3 was used to analyze the knowledge graph and study burst detection [1]. The parameters of CiteSpace were set as follows: time: 1900–2021; interval year: 1; selection criteria: select the top 100 levels with the most citations or occurrences. In the network diagram generated by CiteSpace, nodes represent countries, institutions, cited references, or keywords. When the third node references two nodes together, a link would be created between the two nodes. In co-occurrence network clustering, the clustering module value *Q* was used to evaluate the significance of the modular clustering structure of the network. The greater the network's modularity value, the better the network's clusters. The value interval of *Q* was [0, 1], and *Q* > 0.3 indicates that the clustering structure is significant; S is the average contour value of the cluster, which is used to determine the network's uniformity. It is generally considered that *S* > 0.5 clustering is reasonable. *S* > 0.7 means that the clustering is convincing. VOSviewer 1.6.16 was used to extract the keyword co-occurrence analysis of documents. To simplify the co-occurrence network, we set the co-occurrence threshold to 3 to perform the keywords co-occurrence analysis.

## 3. Results

### 3.1. Distribution of Publication Output

A total of 1109 publications were included in the study. In general, the number of publications of miRNA in OA has been increasing significantly since 2008, as the number of publications increased from 4 in 2008, to 207 in 2020, and 199 in 2021 as of the retrieval date, as shown in Figure 1(a). According to this trend, the total number in 2021 is likely to exceed that in 2020.  Figure 1(b) shows that 78.22% of the total publications are articles and 12.51% of them are reviews, the rest are meeting abstract, early access, proceedings paper, correction and others.  Figure 1(c) shows OSTEOARTHRITIS AND CARTILAGE published the most articles, with 85 publications. There were 34 articles in MOLECULAR MEDICINE REPORTS, 29 articles in INTERNATIONAL JOURNAL OF MOLECULAR SCIENCES, and 26 articles in EXPERIMENTAL AND THERAPEUTIC MEDICINE on miRNAs in OA. The annual citations of publications have been also increased from 11 in 2008 to 5378 in 2020, and 6041 as of 31 October 2021 (Figure 1(d)).

### 3.2. Countries, Institutions, and Authors' Analysis

As shown in Table 1, the country with the most publications was China (690 publications), contributing 58.97% of the total publications, followed by the US (140 publications), England (64 publications), Italy (47 publications), and South Korea (41 publications). Among the top 10 publishing institutions, 6 of them were located in China, 3 in Canada, and 1 in England (Table 1).

In the atlas of institutional cooperation networks, node size represented the number of literature published by countries or institutions, and the connection between nodes reflected the strength of the cooperative relationship. As shown in Figure 2(a), except for the relatively frequent cooperation between the US and Japan, there were few links between different countries and institutions, but within a certain country, there was more cooperation among institutions (Figure 2(b)). The top 20 most prolific authors who published on miRNAs in OA are shown in Table 1, contributed 345 (31.10%) of the total publications. Kapoor M from the University of Toronto had the highest number of publications (30 publications), followed by Wang Y (27 publications), Gandhi R (21 publications), Li J (20 publications), Young DA, and Zhang ZQ (19 publications). 9 of the top 20 most prolific authors are from China. Miyaki S from Hiroshima University had the highest co-citation count (293), followed by Goldring MB (248), Bartel DP (214), Iliopoulos D (189), and Loeser RF (180). As presented in Figure 2(c), prolific authors frequently work in close collaboration with other authors.

### 3.3. Distribution of Co-Cited References

The co-citation network shows the correlation between articles and reflects the knowledge structure of this field. In this study, the top 100 co-cited publications were selected to form a co-citation network. The combined network contains 256,916 references and 65 clusters, 632 nodes, and 3,672 connections. The modular *Q* of the network is 0.6007, indicating that the cluster structure is acceptable. The average contour value is 0.8377, indicating that the network has good uniformity. The labels of the cluster are extracted from the most commonly used headings in the articles of the cluster group. A total of 65 clusters were generated in this network.  Figure 2(d) shows the top 11 largest cluster tags. The cluster tags were #0 chondrogenesis, #1 knee osteoarthritis, #2 ADAMTS5, #3 circular RNA, osteoporosis, #4 apoptosis, #5 DNA methylation, #6 exosomes, #7 bone, #8 MiR-1, #9 embryonic development, and #10 resistin.

We extracted the top 10 co-cited publications and found that Miyaki's article [17] on the dual role of miRNA-140 in chondrogenesis and homeostasis published in Gene & Development in 2010 and Jones's article [18] on the regulation of TNF-*α* and MMP-13 by differentially expressed miRNAs in OA and cartilage tissues were the foundation work of miRNAs in OA research (Table 2).

### 3.4. Co-Occurring Keywords and Cluster Analysis

The analysis of keywords indicates the theme of the publication and the hotspots in the research field. A keyword co-occurrence network composed by the association of these keyword pairs is formed by counting the frequency of the occurrence of keywords in the publications (Figure 3). The frequency of two keywords appearing in the same publication shows the strength between these two keywords. In VOSviewer, we combined keywords with different but identical meanings or singular or plural forms to get a clear network and then classify according to the co-occurrence frequency. A total of 1627 keywords were obtained. In order to simplify the co-occurrence network, keywords with co-occurrence time greater than 3 were selected as the co-occurrence network, and a co-occurrence network composed of 362 keywords was finally obtained (Figure 3). The co-occurrence network has 13 clusters and 7917 connections. The node size in the figure is positively correlated with co-occurrence frequency, and different colors represent different clusters. According to the co-occurrence frequency of keywords, screening and classification were performed (Figure 3), and we found that these publications mainly involved miRNAs, cytokines, signaling pathways, and gene expression. Cytokines involved in the co-occurrence network were IL-1*β*, IL-6, TNF-*α*, TGF-*β*, and MMP-13. The involved signaling pathways and genes included Wnt/*β*-catenin, NF-*κ* B, RUNX2, ADAMTS5, PTEN, SMad4, SIRT1, PI3k/AKT, p53, IRAK1, Bcl-2, C-MYC, and SOX9. The mechanisms involved in OA are apoptosis, proliferation, differentiation, chondrogenesis, degradation, osteogenic differentiation, autophagy, oxidative stress, DNA methylation, inflammation, long noncoding RNA CPG site, and histone deacetylase 4. The cells related to the field of study were cartilage/chondrocyte, mesenchymal stem cells, synovial fibroblast, extracellular matrix, and stromal cell. Furthermore, we found that the chondrocyte was the core of this co-occurrence network (Figure 3), mainly including proliferation, apoptosis, and chondrogenesis, indicating that the function of these miRNAs may be related to chondrocytes and involved the mechanism of cell proliferation and apoptosis.

According to the frequency of occurrence, we combined the repeated miRNAs in the keyword co-occurrence network and found that the number of miRNAs in the network exceeded 100. After merging miRNAs of the same category (merging miR-XA with miR-Xb, miR-XA-3p, and miR-XA-5p), the top 10 miRNAs were miR-140, miR-146, miR-34, miR-181, miR-27, miR-9, miR-29, miR-21, miR-26, and miR-155 (Table 3), suggesting that these miRNAs may be the hotspot miRNAs in this field.

### 3.5. Keywords with Citation Bursts

Burst detection is used to detect keywords that change rapidly in a certain period.  Figure 4 shows the burst keywords in this research area. The blue line indicates the time interval, while the red line indicates the time of the keyword outbreak from start to completion. Keywords with citation bursts first appeared in 2008 (gene), along with the strongest keyword (human articular chondrocyte). The most recent keyword with bursts of citations appeared in 2019 (proliferation, NF-*κ*B, and regeneration). And 4 keywords with citation bursts continue to 2021 (sponge, proliferation, NF-*κ*B, and regeneration). These mutation words reflect the change of research trend in this field in a certain time interval.

## 4. Discussion

### 4.1. Global Description of the Trends of miRNAs in OA Research

According to Figure 1(a), the annual publications of miRNAs in OA research increased rapidly from 2008 to 2020 and after peaked in 2020 to 209, and the publication number is likely to continue increasing in the future based on current trends. This suggested that miRNA has attracted considerable attention in OA research.

The analysis of countries and institutions revealed that Chinese researchers constitute the majority of publications in this area (58.97%, Table 1). This finding could be explained by China's increasing prevalence of OA, which has resulted in a significant increase in demand for health care, which has been complicated by rising healthcare expenses and an aging population (Huibin Long et al.). With the expansion of China's expenditure on OA research, Chinese researchers have shown significant research productivity. However, there was no publication from China in the top 10 highest co-cited publications (Table 2), indicating more work should be done for Chinese researchers. This may be due to being the late mover of this field and the lack of high-quality exploratory research. Meanwhile, Japan occupies the majority of the top 10 most cited publications with a rather small total number of publications [12, 17, 19, 20, 24], indicating that Japanese researchers may play a critical role in the area as well. What's more, the cooperation networks revealed that domestic institutions cooperated frequently, while international cooperation was lacking and needs to be strengthened. Unfortunately, we are not optimistic about future international cooperation under the impact of the global epidemic.

By burst detection in emerging keywords in mRNA research of OA (Figure 4), we found the burst keywords from the beginning of “Genes,” “Rheumatoid Arthritis,” “Tissue.” “Cartilage,” “Differentiation,” and “Human Chondrocytes,” to “Messenger RNA,” “DNA methylation,” “in vitro,” “Gene Expression,” “Transcription Factor,” “Matrix metalloproteinase 13,” “Regulation,” and “NF-*κ*B.” This reflects that the research on miRNAs in OA has gradually begun to focus on the role of tissue cells and molecular mechanisms, and the experimental research methods have shifted from in vivo animal experiments to cell experiments, and from the role of correlation research to molecular mechanism exploration, and the research level has gradually deepened.

### 4.2. The Hotspot miRNAs in OA Research

After merging miRNAs of the same category in the keyword co-occurrence network, we found that the hotspot miRNAs in OA included miR-140, miR-146, miR-21, miR-34, miR-155, miR-203, miR-26, miR-29, miR-125, and miR-141 as shown in Table 3. With different target genes and signaling pathways, they play various roles in early diagnosis, pathogenesis, and potential treatment (Table 3).

MiR-140 is closely related to cartilage homeostasis including chondrocyte proliferation, differentiation, apoptosis, autophagy, and inflammatory responses [26, 27, 29, 53]. In detail, miR-140 is indicated to influence chondrocyte degradation via chondrogenic factor transcription factor SRY-box-containing gene 9 (SOX9), ADAMTS, fucosyltransferase (FUT), and runt-related transcription factor (Runx2) regulators and pathways [26, 27, 29, 53]. Furthermore, miR-140 plays a critical role in E2-mediated cartilage homeostasis, as it allows E2 to suppress the production of MMP-13, thereby protecting chondrocytes from degradation [30]. Therefore, miR-140 could be a target for OA therapeutic interventions.

MiR-146a, as the main member of the miR-146 family, is found promoting chondrocyte autophagy through Bcl-2, which is induced by hypoxia [31]. It also promotes chondrocyte apoptosis by increasing the level of vascular endothelial growth factor (VEGF) in cartilage via Smad4 [33] and participates in inflammation [54]. Additionally, miR-146a is inferred regulating MMP-13 through IRAK1, TLR4, and TRAF6 to maintain the delicate balance of ECM homeostasis [34].

MiR-34 promotes chondrocyte death and OA progression via DLL1 and PI3K/AKT pathway modulation [36]. Similarly, earlier research has demonstrated that silencing miR-34a with LNA-modified antisense can significantly inhibit rat chondrocyte apoptosis produced by IL-1*β* [36]. Additionally, miR-34a-5p has been shown to affect chondrocyte proliferation, autophagy, and apoptosis by targeting SYVN1 [37], providing a novel insight into the OA pathogenesis.

MiR-181 could be a potential biomarker to screen OA patients [51]; it also upregulates caspase-3, PARP, MMP-2, and MMP-9 expression, inhibiting cell proliferation and promoting apoptosis in OA chondrocytes via PTEN targeting [38]. Furthermore, the study found that decreasing miR-181 expression can lower the inflammatory factors TNF-*α* and IL-6 expression by downregulating the NF-*κ*B signaling pathway, thereby suppressing the occurrence of OA [39].

MiR-27 upregulation inhibits OA pathogenesis through targeting leptin and inhibiting the NF-*κ*B signaling pathway [40]. It exerts protective effects against OA. MiR-27 is also thought to be a target of lncRNA-CIR and MMP-13, both of which are involved in chondrocyte extracellular matrix (ECM) degradation in OA [27, 41].

MiR-9 is a potential therapeutic target for OA. Exosomal miR-9-5p, which is secreted by bone marrow-derived mesenchymal stem cells, has been shown to alleviate OA by inhibiting syndecan-1 [42]. And inhibition of LncRNA MIR22HG ameliorated IL-1*β*-induced apoptosis and ECM degradation of human chondrocytes through miR-9-3p/ADAMTS5 pathway (Hui Long et al.). Furthermore, resveratrol is also reported to have a therapeutic effect in OA by regulating the MALAT1/miR-9/NF-*κ*B signaling pathway [43].

The miR-29 family negatively regulated SMAD, NF-*κ*B, and canonical WNT signaling pathways, and they are also regulated by TGF-*β*1 and IL-1 in chondrocytes [44]. WNT-related genes, such as FZD3, FZD5, DVL3, FRAT2, and CK2A2, are validated as direct targets of the miR-29 family. Moreover, miR-29b-3p promotes chondrocyte apoptosis and facilitates the occurrence and development of OA by targeting PGRN [45]. And Bax targeted by miR-29a regulates chondrocyte apoptosis as well [46].

MiR-21 is identified as a regulator of growth arrest-specific 5 (GAS5) during OA pathogenesis, by increasing the expression levels of MMPs, thus stimulating apoptosis and suppressing autophagic responses [47]. Likewise, miR-21-5p promotes hyaline cartilage production, protecting IL-1*β*-induced chondrocytes from degradation [48], and regulates ECM degradation and angiogenesis by targeting Spry1 [49]. Moreover, the recent study showed that the novel NF-*κ*B inhibitor sc75741 mitigates chondrocyte degradation and prevents activated fibroblast transformation by modulating miR-21/gdf-5/sox5 signaling [55], which may be a potential treatment for OA.

MiR-26a and miR-26b mediate OA progression by targeting FUT4 via the NF-*κ*B signaling pathway [52]. Furthermore, miR-26a reduces cartilage injury and synovial inflammation in OA of knee joints by inhibiting the activation of the NF-B signaling pathway [56].

It has been shown that miR-155 plays an important role in chondrocyte degradation via the upstream MAPK pathway. Furthermore, recent studies indicate that frugoside (FGS) inhibits macrophage M1 polarization by partially downregulating miR-155 levels, so decreasing IL-6 and TNF-*α* secretion, thereby delaying ECM and cartilage degradation and chondrocyte hypertrophy [50]. Besides, exosomes produced from synovial mesenchymal stem cells overexpressing miR-155-5p prevent OA by promoting proliferation and migration, inhibiting apoptosis, and regulating ECM secretion in chondrocytes. Therefore, miR-155 is most likely a potential OA therapeutic target [50].

### 4.3. Chondrocytes are Potential Targets for Most miRNAs in OA

According to the keywords co-occurrence network, chondrocytes are most closely linked to miRNAs in the research field of OA, as well as the core elements of the co-occurrence network. Chondrocytes are responsible for synthesizing ECM components and maintaining cartilage homeostasis. A strong relationship between miRNAs and chondrocytes has been reported in prior studies. The top 10 miRNAs we found were also closely related to chondrocytes. They mainly correlate with the apoptosis, degradation, autophagy, proliferation, and differentiation of chondrocytes. In detail, most of the miRNAs in the list are found to promote chondrocyte apoptosis and exacerbates the progression of OA, while miR-140 is essential for normal endochondral bone development, accelerating chondrocyte proliferation and differentiation [16, 57]. Furthermore, miR-140 and miR-34a are closely involved in the dynamic balance between proliferation and apoptosis of chondrocytes, thus maintaining the stability of cartilage quantity and function [18, 32]. Meanwhile, due to the protective and antiapoptotic functions of chondrocyte autophagy [28, 54], miRNAs like miR-146 [58] and miR-155 [59] regulate the expression of the autophagy-associated gene (ATG) in chondrocytes during this process to balance of material and energy metabolism of chondrocytes.

Moreover, the pathology of MMP transcription concerning proinflammatory cytokines as IL-1*β*, IL-6, TNF-*α*, TGF-*β*, and NF-*κ*B was also involved in the co-occurrence network. Much of the literature we retrieved on miRNAs in OA showed that miR-140, miR-146a, miR-155, and miR-124 can mediate MMP-13 through TNF-*α*, IL-1*β*, and NF-*κ*B, which may affect chondrocyte degradation. The keywords co-occurrence network includes involving signaling pathways and genes Wnt/*β*-catenin, NF-*κ*B, RUNX2, ADAMTS5, PTEN, SMad4, SIRT1, PI3k/AKT, p53, IRAK1, Bcl-2, C-MYC, and SOX9.

## 5. Strengths and Limitations

Our study used bibliometric and visual analyses to assess the status and trends of miRNA research in OA. The following limitations, however, must be mentioned. The data were retrieved only from the databases of the Web of Science, and other databases like PubMed, MEDLINE, EMBASE, and Google Scholar were not included. Although we found that China was the leading country in the total number of publications, we did not have data from major Chinese databases like the China National Knowledge Infrastructure Database (CNKI), Wanfang Data Journal Database, Chinese Biomedical Literature Database, and Chongqing VIP database. And the limited terms were used in the publication retrieval strategy, so we may not have identified all the relevant studies in the field. Furthermore, differences between the real world and the current results may exist. For example, different literature types may cause bias to our study because reviews may have higher citations than original studies. Additionally, some recently published high-quality papers might not be highlighted due to low citation frequency for the short time in publication.

## 6. Conclusion

This study showed the current status and global trends of miRNAs in OA research. Furthermore, the study showed miR-140, miR-146, miR-34, miR-181, miR-27, miR-9, miR-29, miR-21, miR-26, and miR-155 were hotspot miRNAs in OA; besides, chondrocytes could be a potential target for OA treatment. More studies should be focused on the relationship between miRNAs and chondrocytes in the future [17, 60–64].

## Figures and Tables

**Figure 1:** Citation of publications related to osteoarthritis. (a) The number of annual publications till 2021, (b) types of publications, (c) number of publications having osteoarthritis with most citations in different journals, and (d) the annual citations of publications till 2021 with osteoarthritis.

**Figure 2:** Literature published by countries and institutions regarding OA. (a) Relative cooperation and links between countries for publications in the same area, (b) relative cooperation and links between different institutions for publications in the same area in China, (c) prolific authors frequently work in close collaboration with other authors, and (d) most commonly used headings in articles, which were used as labels in the cluster network.

**Figure 3:** Co-occurring keywords and cluster analysis of reported literature.

**Figure 4:** Keywords with citation bursts.

**Table 1:** Countries, institutions, and authors' analysis.

Country	Publications (%)	Institution	Publications (%)	Author	Publications	Cited author	Counts
China	690 (58.97%)	Sun Yat-sen University	40 (3.61%)	Kapoor M	30	Miyaki S	293
United States	140 (12.62%)	Xi'an Jiaotong University	34 (3.07%)	Wang Y	27	Goldring MB	248
England	64 (5.77%)	University of Toronto	33 (2.98%)	Gandhi R	21	Bartel DP	214
Italy	47 (4.24%)	Shanghai Jiaotong University	30 (2.71%)	Li J	20	Iliopoulos D	189
South Korea	41 (3.70%)	University Health Network Toronto	30 (2.71%)	Young DA	19	Loeser RF	180
Japan	39 (3.52%)	Krembil Research Institute	29 (2.61%)	Zhang ZQ	19	Akhtar N	154
Canada	39 (3.52%)	Newcastle University UK	24 (2.16%)	Kang Y	18	Jones SW	154
Germany	20 (1.80%)	Jilin University	23 (2.07%)	Zhang Y	18	Yamasaki K	148
Spain	18 (1.62%)	Nanjing Medical University	22 (1.98%)	Barter MJ	16	Swingler TE	128
Netherland	18 (1.62%)	Shandong University	22 (1.98%)	Clark IM	16	Song J	125

**Table 2:** Distribution of co-cited references of the published articles.

Rank	Co-cited publications	First author (year)	Counts
1	MicroRNA-140 plays dual roles in both cartilage development and homeostasis [17]	Miyaki S (2010)	113
2	The identification of differentially expressed microRNA in osteoarthritic tissue that modulates the production of TNF-alpha and MMP-13 [18]	Jones SW (2009)	101
3	MicroRNA-27b regulates the expression of matrix metalloproteinase 13 in human osteoarthritis chondrocytes [19]	Akhtar N (2010)	98
4	Macro view of microRNA function in osteoarthritis [12]	Miyaki S (2012)	96
5	MicroRNA-140 is expressed in differentiated human articular chondrocytes and modulates interleukin-1 responses [20]	Miyaki S (2009)	95
6	Integrative microRNA and proteomic approaches identify novel osteoarthritis genes and their collaborative metabolic and inflammatory networks [21]	Iliopoulos D (2008)	88
7	Characterization of microRNA expression profiles in normal and osteoarthritic human chondrocytes [22]	Diaz-Prado S (2012)	88
8	The expression and function of microRNAs in chondrogenesis and osteoarthritis [23]	Swingler TE (2012)	87
9	Expression of microRNA-146a in osteoarthritis cartilage [24]	Yamasaki K (2009)	86
10	Osteoarthritis: a disease of the joint as an organ [25]	Loeser R. (2012)	76

**Table 3:** Different pathways and their function.

miRNAs	Frequency (Strength)		Pathways (Genes)	Functions
**miR-140**	**12** (99)	miR-140 [23–26]	SOX9/ADAMTS5/FUT/RUNX2	↑chondrocyteproliferation/differentiation
		miR-140 [27]	E2/MMP-13	↓chondrocyte apoptosis/autophagy
		miR-140 [28]	ADAMTS5/TIMP1/SP1/MMP13	↓chondrocyte degradation
				↓matrix degradation
**miR-146**	**4** (30)	miR-146a [29]	Bcl-2	↑chondrocyte autophagy
		miR-146a [30]	VEGF /SMAD4/TGF-b	↑chondrocyte apoptosis
		miR-146a [31]	TLR4/TRAF6/IRAK1/MMP-13	↓ECM homeostasis
		miR-146a [32]	IRAK1/TRAF6	↑Inflammation
**miR-34**	**6 (42)**	miR-34 [65]	DLL1/PI3K/AKT	↑chondrocyte apoptosis
		miR-34a [33]	IL-1*β*	↑chondrocyte apoptosis
		miR-34a-5p [34]	SYVN1	↑chondrocyte proliferation/apoptosis/autophagy
**miR-181**	**5 (42)**	mir-181 [35]	PTEN/Caspase-3/PARP/MMP-2/MMP-9	↓cell proliferation ↑chondrocyte apoptosis
		mir-181 [36]	NF-*κ*B/TNF-*α*/IL-6	↑inflammatory
**miR-27**	**4 (32)**	miR‐27 [37]	NF-*κ*B/IL-6/IL-8	↓inflammatory
		miR‐27‐3p/miR-27b [38, 39]	MMP13	↓ECM degradation ↓chondrocyteapoptosis
**miR-9**	**4 (33)**	miR-9-5p [40]	SDC1	↓Inflammatory ↓oxidative stress injury
		miR-9-3p [41]	ADAMTS5/IL-1*β*	↓apoptosis ↓ECM degradation
		miR‑9 [42]	MALAT1/NF‑*κ*B	↑chondrocyte's growth
**miR-29**	**3 (25)**	miR-29 [43]	SMAD/NF-*κ*B/WNT/TGF-*β*1/IL-1	↑chondrocyte apoptosis
		miR-29b-3p [44]	PGRN	↑chondrocyte apoptosis
		miR-29a [45]	BAX	↑chondrocyte apoptosis
**miR-21**	**3 (27)**	miR-21 [46]	GAS5/MMPs	↑chondrocyte apoptosis ↓chondrocyte autophagy
		miR-21-5p [47]	IL-1*β*	↑chondrocyte degradation
		mir-21 [48, 49]	Spry1/ GDF-5/SOX5/NF-*κ*B	↑chondrocyte degradation ↑angiogenesis
**miR-26**	**2 (18)**	miR-26a/26b [50, 51]	FUT4/NF-*κ*B	↓inflammatory ↓cartilage injury
**miR-155**	**2 (18)**	miR-155 [51]	NF-*κ*B/JNK AP-1/MMP-13	↑chondrocyte degradation
		miR-155-5p [52]	IL‐6/TNF‐*α*	↑chondrocyte degradation and hypertrophy

## Data Availability

Data will be provided upon request to the authors.
